# Preoperative Prediction of Axillary Lymph Node Metastasis in Breast Cancer Based on Intratumoral and Peritumoral DCE-MRI Radiomics Nomogram

**DOI:** 10.1155/2022/6729473

**Published:** 2022-08-18

**Authors:** Ying Liu, Xing Li, Lina Zhu, Zhiwei Zhao, Tuan Wang, Xi Zhang, Bing Cai, Li Li, Mingrui Ma, Xiaojian Ma, Jie Ming

**Affiliations:** ^1^Special Needs Comprehensive Department, Affiliated Tumor Hospital of Xinjiang Medical University, Urumqi 830011, Xinjiang, China; ^2^Medical Imaging Center, Affiliated Tumor Hospital of Xinjiang Medical University, Urumqi 830011, Xinjiang, China; ^3^Information Center, Affiliated Tumor Hospital of Xinjiang Medical University, Urumqi 830011, Xinjiang, China; ^4^Medical Imaging Center, Bachu County People's Hospital, Bachu 843800, Xinjiang, China

## Abstract

**Objective:**

To investigate the value of preoperative prediction of breast cancer axillary lymph node metastasis based on intratumoral and peritumoral dynamic contrast enhancement magnetic resonance imaging (DCE-MRI) radiomics nomogram. *Material and Methods*. In this study, a radiomics model was developed based on a training cohort involving 250 patients with breast cancer (BC) who had undergone axillary lymph node (ALN) dissection between June 2019 and January 2021. The intratumoral and peritumoral radiomics features were extracted from the second postcontrast images of DCE-MRI. Based on filtered radiomics features, the radiomics signature was built by using the least absolute shrinkage and selection operator method. The Support Vector Machines (SVM) learning algorithm was used to construct intratumoral, periatumoral, and intratumoral combined periatumoral models for predicting axillary lymph node metastasis (ALNM) in BC. Nomogram performance was determined by its discrimination, calibration, and clinical value. Multivariable logistic regression was adopted to establish a radiomics nomogram.

**Results:**

The intratumoral combined peritumoral radiomics signature, which was composed of fifteen ALN status-related features, showed the best predictive performance and was associated with ALNM in both the training and validation cohorts (*P* < 0.001). The prediction efficiency of the intratumoral combined peritumoral radiomics model was higher than that of the intratumoral radiomics model and the peritumoral radiomics model. The AUCs of the training and verification cohorts were 0.867 and 0.785, respectively. The radiomics nomogram, which incorporated the radiomics signature, MR-reported ALN status, and MR-reported maximum diameter of the lesion, showed good calibration and discrimination in the training (AUC = 0.872) and validation cohorts (AUC = 0.863).

**Conclusion:**

The intratumoral combined peritumoral radiomics model derived from DCE-MRI showed great predictive value for ALNM and may help to improve clinical decision-making for BC.

## 1. Introduction

Breast cancer (BC) is the most common malignant tumor in females, and the 5-year relative survival rate of patients with BC is as high as 98.6% [1, 2]. However, the survival rate decreases to 84.4% in BC patients with regional axillary lymph node metastasis (ALNM) [3]. Axillary lymph node (ALN) status is important for tumor staging, treatment decisions, and prognosis of patients with BC [4, 5]. ALN status is the most important prognostic factor affecting local recurrence and long-term overall survival of BC [6]. Sentinel lymph node biopsy (SLNB) is the main means for diagnosis of sentinel lymph node metastasis (SLNM). Once SLNM is confirmed after SLNB, axillary lymph node dissection (ALND) is performed to confirm the staging. However, a prior study found [7] that nearly half of the patients had metastasis in SLNs, but no metastasis in non-SLNs, and ALND is not necessary among all patients with SLNs. For patients with only SLNM, the significance of ALND is only to clarify the axillary stage. In terms of treatment, for patients with SLNM, up to 40%–70% of treatments for ALND are meaningless [8]. Hence, the preoperative noninvasive prediction of ALN status is extremely important.

Dynamic contrast-enhanced magnetic resonance imaging (DCE-MRI) plays an increasingly important role in identifying ALNM. DCE-MRI provides a set of high-quality images from the lesion, including useful information not only about the shape and boundary but also about the dynamic behavior of the contrast agent in the lesion [9, 10]. Moreover, DCE-MRI and its parameters are used to reflect tumor angiogenesis and the internal microenvironment [11].

Radiomics transforms digital medical images into mineable data by high-throughput extraction of rich quantitative image features based on shape, intensity, size, and volume [12]. The application of these data in clinical decision support can provide better diagnosis, prognosis, and prediction accuracy [13, 14]. The association between intratumor heterogeneity and metastatic spread was identified in a previous study [15]. Several studies [16–19] used image-based methods for the preoperative prediction of ALN metastasis in BC, colorectal cancer, bladder cancer, and lung adenocarcinoma and achieved good prediction results. However, previous studies mostly focused on disease information reflected by the external contour information of the lesion without noticing the potential value of the internal imaging features of the tumor. The purpose of this study was to investigate and verify the value of a DCE-MRI intratumoral combined with a peritumoral radiomics nomogram in the preoperative prediction of the ALN status of BC.

## 2. Information and Methodology

### 2.1. Subjects of Study

Retrospective analysis of clinical, pathological, and MRI data of 312 patients with BC confirmed by surgery or biopsy pathology from June 2019 to January 2021 at the Affiliated Cancer Hospital of Xinjiang Medical University, including 291 cases of invasive ductal carcinoma, 6 cases of invasive lobular carcinoma, and 15 cases of papillary carcinoma. The age range of patients was 26∼79 years, with a mean age of 49.0 ± 9.7 years. The patients were divided into the ALN-positive cohort (*n* = 190) and the ALN-negative cohort (*n* = 122) based on ALN pathological findings. Random sampling was used to split the patients into 250 cases in the training cohort and 62 cases in the validation cohort according to a ratio of 8 : 2. The study was approved by the Medical Ethics Committee of the Affiliated Cancer Hospital of Xinjiang Medical University (approval number: K2021028), and subjects were exempted from informed consent.

### 2.2. Inclusion Criteria and Exclusion Criteria

Inclusion criteria: (i) adult females aged 18 years and older; (ii) confirmed BC by histopathology; (iii) patients who underwent mammography or surgical pathology biopsy one week after breast MR examination and underwent ALNB or ALND; (iv) patients who had not been diagnosed with any other cancers. Exclusion criteria: (i) patients who have undergone previous breast puncture, surgery, radiotherapy, chemotherapy, or hormone therapy; (ii) patients who reported incomplete clinical or pathological data; (iii) patients who have been diagnosed with nonlumpy BC; (iv) poor quality MRI images that cannot be evaluated. The clinical data, including age, menopausal status, MR-reported maximum diameter of the lesion, and MR-reported ALN status, were collected from all cases. Our research flow chart is shown in Figure 1.

### 2.3. MRI Examination Methods

The examination equipment was a Siemens Verio Tim 3.0 T superconducting MR scanner (Siemens Healthiness, Erlangen, Germany) and an 8-channel breast phased-array coil. The patients were asked to remain in a prone position with bilateral mammary glands placed naturally down in the coil and strictly braked. The scans were as follows: the bilateral breast was the anterior post, with the anterior part of the thorax at the same level. All patients underwent plain breast MRI and multiphase dynamic enhancement scans. Standard imaging was performed: DCE-MRI applied an axial three-dimensional fluid-attenuated inversion recovery (3D-FLAIR) sequence. Plain and contrast-enhanced scans were acquired for all patients. The enhancement scan was conducted by the following parameters: flip angle of 10°; slice thickness 1.2 mm; 0.2 mm gap; field of view (FOV) 340 × 340 mm; matrix 448 × 336 mm. Gadolinium with diethylenetriamine pentaacetic acid (Gd-DTPA) was injected into the dorsal hand vein with a high-pressure syringe at a dose of 0.2 mL/kg at a rate of 2.5 mL/s. Twenty milliliters of saline was injected at the same rate in the cohort after the contrast injection. The scan was started immediately after the injection, and seven consecutive periods of 1 min each were scanned.

### 2.4. MRI Image Acquisition and Radiological Evaluation

Breast MRI images of all enrolled patients were extracted from the picture archiving and communication system (PACS) in digital imaging and communications in medicine (DICOM) format. Two experienced radiologists reviewed all MR scan images to evaluate the following traits for each BC patient: (i) maximum diameter of the tumor was defined as the maximum diameter on the transverse image; (ii) positive ALNM was defined as a shorter axis diameter greater than 10 mm or central necrosis. The radiologists were told about the BC diagnosis but not the clinical and pathological details, and they would keep readings for 14 consecutive days. Disagreements were resolved through consultation.

### 2.5. Region-of-Interest (ROI) Segmentation and Radiation Feature Extraction

The incoming breast DCE-MRI images were exported from the PACS system in DICOM format, and the second postcontrast images of DCE-MRI were imported into 3D-Slicer software (version 4.11). ROI profiling was performed by two senior physicians with 15 and 12 years of experience in breast MR imaging diagnostics to manually map the intratumoral region along the edge of the tumor layer by layer, and the circum tumor region (5 mm of extravasation) was automatically mapped by software to construct the total volume of interest (VOI). Avoiding necrosis of the tumor, if the breast skin or chest wall was less than the maximum distance from the tumor circumference, the breast skin surface or chest wall to the tumor circumference was determined to be the maximum distance. Multicentre and multifocal cases were selected for the largest lesions. Pyramidimocs software was used to extract the intratumoral and peritumoral radiomics features.

### 2.6. Radiation Feature Selection and Signature Construction

We devised a three-step program for dimensional reduction and robust feature selection. First, the ROI segmentation was performed in a blinded fashion by one radiologist (reader XL) and another radiologist (reader 2, LNZ); both radiologists were aware of the diagnosis of BC but were blinded to the clinical and pathologic details. Intraclass correlation coefficients (ICCs) were calculated to evaluate the reliability and reproducibility of features by using 60 randomly chosen MR images. Radiomics features with ICC > 0.75 (excellent stability) were used for feature extraction [20]. Second, all feature lines were standardized by the *z* score standardization method, and the correlation between features was calculated by the Spearman correlation coefficient. For features with a correlation coefficient >0.9, one of the two features was retained. Third, the least absolute shrinkage and selection operator logistic regression algorithm, with penalty parameter tuning conducted by 10-fold cross-validation, was then applied to select ALN-status-related features with nonzero coefficients from the training cohort. A radiomics signature was generated by a linear combination of selected features weighted by their respective coefficients.

### 2.7. Establishment Performance and Validation of the Radiodiomic Model

The Support Vector Machines (SVM) learning algorithm was used to establish a prediction model for ALN metastasis in the training cohort, and the diagnostic accuracy, sensitivity, and specificity indices derived from the confounding matrix and its derivations were used to evaluate the diagnostic efficacy of all three models. Univariate logistic regression analysis was performed to screen independent predictors of ALN status in patients with BC with age, menopausal status, radiomics signature, MR-reported maximum diameter of the disease, and MR-reported ALN status. A radiomics nomogram was established in combination with a radiomics signature and independent prognostic factors. The diagnostic efficacy of the radiomics nomogram was validated in the validation cohorts, and ROC curves were drawn to evaluate the diagnostic efficacy of the nomogram [21, 22]. The calibration efficiency of the nomogram was evaluated by drawing calibration curves, and Hosmer-Lemes showed that analytical fit was used to evaluate the calibration ability of the nomogram. Mapping decision curve analysis (DCA) was performed to evaluate the clinical utility of the predictive models.

### 2.8. Statistical Analysis

Using Python (3.7.13), normally distributed measurements were expressed as $\bar{x}$ ± *s* in mean numbers, and two independent sample *T* assays were used for comparison between the two cohorts. Nonconforming measurements were expressed as medians (upper and lower quartiles), and two independent Mann–Whitney *U*-rank sum tests were used for comparisons between the two cohorts. Count data are expressed in *n* (%), and *χ*^2^ assays were used to compare the two cohorts. All *P* values were bilateral assays with a statistically significant difference of *P* < 0.05.

## 3. Results

### 3.1. Patient Clinical, MR Data

The clinical and MR imaging data of patients in the training cohort and the validation cohort are shown in Table 1. The rates of ALN metastasis were 39.2% (98/250) and 38.7% (24/63) in the training and validation cohorts, respectively, whereas no difference was found between cohorts (*P* > 0.05). In total, 50 patients (24.0%; 50/208) with ALN metastasis were understaged, and 32 patients (30.8%; 32/104) without ALN metastasis were overstaged according to ALN status reported at MR. The overall diagnostic accuracy of the subjective MR report of ALN status was 230 of 312 (73.7%), with a sensitivity of 72 of 122 (59.0%), a specificity of 158 of 190 (83.2%), a positive predictive value of 72 of 104 (69.2%), and a negative predictive value of 158 of 208 (76.0%).

### 3.2. Feature Selection and Construction of Radiomics Signature

In patients with BC, each intratumoral and peritumoral VOI was extracted from 1906 radiomics features. An early fusion was used to combine all features into 3812 radiomics features extracted from DCE-MRI phase 2 images of intratumoral, peritumoral, and intratumoral combined with peritumoral DCE-MRI. Feature screening using minimal absolute contraction and selection of operator logistic regression models was performed in the training cohort (Figure 2) to obtain 12, 7, and 15 ALN state-related features with nonzero coefficients for subsequent analysis. The greater the absolute value of the characteristic regression coefficient, the greater the correlation with ALN status in BC and the higher the predictive value. The radiomics signature was constructed, and the intratumoral combined peritumoral radiomics score was calculated by using the following formula:intratumoral combined peritumoral radiomics score = 0.40041734218938885 + 0.016776*∗*lbp-3D-k_first order_Skewness + 0.011962*∗*lbp-3D-k_glcm_Imc2 + 0.036346*∗* lbp-3D-m2_glcm_ClusterShade_x-0.047465*∗*log-sigma-3-0-mm-3D_firstorder_10Percentile_x-0.006153*∗*wavelet-HHL_firstorder_Kurtosis_x-0.027324*∗*wavelet-HLH_glcm_ Idm-0.019761*∗*wavelet-HLH_glcm_Idn + 0.000874*∗*wavelet-LHL_glcm_Correlation+0.049144*∗*gradient_firstorder_ Skewness-0.022611*∗*log-sigma-3-0-mm-3D_glrlm_GrayLevelVariance_y-0.007552*∗*square_glszm_GrayLevel Variance-0.015879*∗*wavelet-LHH_glszm_GrayLevelVariance_y-0.003411*∗*wavelet-LHL_firstorder_Skewness_*y* (Note: Suffixes are the hallmarks of *y*, all of which are tumour circumference). Detailed information on the formula for intratumoral combined with peritumoral radiomics score is presented in the Appendix.

### 3.3. Establishment, Performance, and Validation of Predictive Models

ROC curves were used to evaluate the prognostic efficacy of three imaging models of intratumoral, peritumoral, and intratumoral combined with peritumoral in the training cohort and the validation cohort for BC ALN status. The results suggest that intratumoral combined with peritumoral models were more predictive than intratumoral or peritumoral models, as shown in Table 2.

Furthermore, after Wilcoxon assays, the intratumoral combined with peritumoral radiomics signature in patients with ALN metastasis was higher in the training and validation cohorts than in the nonmetastatic cohorts, with statistically significant differences between cohorts (*P* < 0.001). Therefore, intratumoral combined with peritumoral models were selected for radiomics nomogram later in this study. A radiomics nomogram (Figure 3(a)) incorporated three independent predictors (radiomics signature, MR-reported ALN status, and MR-reported MaxDiameter). All prediction model receiver operating characteristic curves are provided in Figures 3(b) and 3(d). In the training and validation cohorts, the radiomics nomogram showed the highest discrimination between positive and negative for ALN metastasis, with AUCs of 0.872 (95% CI: 0.829, 0.915) and 0.863 (95% CI: 0.770, 0.956); the observed AUC value was higher than that of the intratumoral combined with the peritumoral radiomics model, intratumoral radiomics model, peritumoral radiomics model,1 and MR-reported ALN status alone. Nomogram calibration curves (Figures 3(c) and 3(e)) showed good agreement between the predicted and observed axillary lymph node metastasis training cohorts and the validation cohort. The *P* values of the Hosmer-Leme test were 0.97 and 0.62, respectively. This shows that the nomogram fits perfectly in both the training and validation cohorts.

### 3.4. Clinical Benefit

The decision curve analysis for the radiomics nomogram, the intratumoral model, the periatumoral model, and intratumoral combined with periatumoral model are presented in Figure 4. Compared with scenarios in which no prediction model would be used (i.e., treat-all or treat-none scheme), radiomics nomogram showed significant benefit for intervention in patients with a prediction probability of 17%–77% compared to intratumoral (23%–54%), peritumoral (24%–52%), intratumoral combined with peritumoral (22%–65%), and the yield was also higher than other radiomics models. Preoperative prediction of axillary lymph node status in BC using a radiomics nomogram with intratumoral combined with a peritumoral radiomics signature has better clinical benefit. The diagnostic efficiency of the radiomics nomogram (AUC = 0.863) was higher than that of senior radiologists (AUC = 0.775). The difference in AUC was statistically significant by Delong (*P* < 0.001), so the radiomics nomogram has a good clinical application value.

## 4. Discussion

ALNM is not only an important prognostic factor for BC but also a key indicator for determining the stage and guiding treatment of this disease [23]. The present study developed and validated a radiomics nomogram that was constructed by the intratumoral combined peritumoral radiomics signature, the MR-reported maximum lesion diameter, and the MR-reported ALN status. When used for noninvasively predicting the ALN status of patients with BC before surgery, this nomogram showed great differential diagnosis in both the training cohort (AUC = 0.872) and validation cohort (AUC = 0.863) and had better performance than that of both the simple radiomics model and experienced MR diagnostic doctors.

Prior studies have shown that the tumor microenvironment contains multiple immune cells, blood vessels, and extracellular matrix and that alterations in immune cell distribution and angiogenesis may promote tumor development and metastasis.

However, ALN metastasis is diagnosed based on MR showing that the diameter of the short axis of the axillary lymph node is greater than 10 mm or that there is a necrotic area in the center of the axillary lymph node. The present study shows that the accuracy, sensitivity, and specificity of MR reports in diagnosing ALN metastasis are 73.7%, 59.0%, and 83.2%, respectively. A considerable proportion of patients could be misclassified according to the macro appearance of ALN images, consistent with several previous studies [24, 25]. It has been reported that metastatic ALNs accounted for 80.77% of ALNs with short diameters ≥10 mm and 45.28% of ALNs with short diameters of 4–9 mm [26]. Therefore, traditional imaging tests are of limited value in assessing changes in the tumor microenvironment, especially in predicting ALN status in early BC with no changes in size, morphology, and signal but infiltration of cancer cells. Similarly, it remains challenging to distinguish benign and malignant ALNs based only on the morphological characteristics or metabolic activity of ALNs [27, 28].

MRI can accurately measure lesion size, and there is no significant difference between the pathological findings and results. This was also found in the present study, which may be associated with robust growth and metabolism in larger lesions, consistent with KIM and others [29]. We found that, as independent predictors of BC ALNM, MR-reported maximum lesion diameter and MR-reported ALN status significantly improved the model's predictive efficacy, although they had a small contribution weight to the radiomics nomogram. In addition, the AUCs of the other two factors for the intratumoral combined peritumoral prediction model increased from 0.867 to 0.872 in the training cohort and from 0.785 to 0.863 in the validation cohort.

In this study, the nomogram with the best diagnostic efficiency included 13 intratumoral and 2 periatumoral radiomics features. These 13 intratumoral features consist of 9 texture features and density features, and both periatumoral features are density features. The texture features describe the quantization of grey changes in the image region, which has rotation invariance and strong antinoise ability and is greatly affected by resolution density features. It is also known as grey histogram information, which can simply describe the global distribution of grey in an image and have rotation invariance. Although these data cannot be used for humans to perceive, they are predictive of tumor status and are easily captured by radiomics analysis. In this study, there were statistically significant differences in texture and density between the positive and negative ALNM cohorts, which might be due to local density and texture heterogeneity due to tumor heterogeneity and malignancy between the two cohorts.

The heterogeneity of BC mainly originates from heterogeneity within tumors and the heterogeneity of the microenvironment around tumors. Some features of the tumor microenvironment may be the driving forces of cancer progression, metastasis, and initiation of treatment resistance [30–32]. Macrophages and fibroblasts are the most common cells in the BC microenvironment and contribute to ALNM in BC. They can regulate the construction of the extracellular matrix and proliferation and migration of BC cells and then influence the survival of BC [33]. The literature has shown that normal tissues around the training tumor will also be affected by cancer cells with tumor invasion or metastasis [34]. It is possible to capture the heterogeneity and complexity of the tumor microenvironment by extracting the imaging features of peritumoral tissue to better assess its biological behavior and conduct an early intervention. To distinguish lung polyps from nonsmall cell lung cancer, Beig et al. [35] extracted the imaging features of lung nodules and 30 mm outside the nodules. Its predicted performance AUC was improved from 0.74 to 0.80. [36] evaluated whether pathological complete response (PCR) can be obtained after neoadjuvant chemotherapy in BC by using the DCE-MRI imaging radiomics features in peritumor and inside the tumour, and the results showed that the combination of peritumoral and intratumoral imaging features of 2.5 mm to 5.0 mm outside the tumor could predict the ability to obtain PCR in patients with BC, providing a theoretical basis for the selection of BC treatment. This study referred to the peripheral tumor area defined by Braman *et al.* With the imaging features extracted from the 5.0 mm peritumor of BC, the AUCs of intratumoral, peritumoral, and intratumoral combined with peritumoral models for predicting ALNM of BC were 0.844, 0.828, and 0.867 in the training cohort and 0.708, 0.616, and 0.785 in the validation cohort, respectively. These data suggest that the peritumoral features of DCE-MRI contain valuable information about tumor metastasis, which should be included in further imaging studies.

This study analyzed the radiomics features of phase II DCE-MRI of three-dimensional lesions of BC. DCE-MRI can provide images with high time, high space, and high signal-to-noise ratio by evaluating tumor morphology and hemodynamics to diagnose breast diseases. Phase II images are significantly enhanced and can better reflect the aggressiveness and heterogeneity of tumors. Three-dimensional lesions can also comprehensively reflect the overall situation and heterogeneity of the tumor. It is of great value to focus on more MRI sequences in subsequent studies, and it could be expected that the multimodal MRI image radiomics model could provide us with more useful information and that the prediction efficiency of the model could be further improved.

This study also has certain limitations. First, this is a single-center and small-sample retrospective study, and the external validation of the stability and clinical applicability of the model needs to be added to a multicentre dataset in the future. Second, the outline of the BC lesion VOI is a semiautomatic outline, and the boundary of the lesion is confirmed manually, which is time-consuming. However, the current gold standard for segmenting images is still a manual outline based on physician experience, and the outliner more mature artificial intelligence automatic segmentation algorithms are to be developed and applied to improve segmentation efficiency and reduce subjective inconsistency. Finally, only radiomics features derived from the second postcontrast images of DCE-MRI were analyzed due to their crucial role in the diagnostic performance of breast MRI. Hence, other DCE-MRI series deserve to be investigated in further studies.

## 5. Conclusion

We propose a noninvasive and convenient imaging radiomics nomogram that combines the radiomics signature, MR-reported maximum lesion diameter, and MR-reported ALN status for the preoperative evaluation of ALN status in patients with BC. It provides more reliable reference information for prognosis judgment and clinical decision-making.

## Figures and Tables

**Figure 1:** Workflows for the necessary steps in the current study. Layer-by-layer manual segmentation of tumors was performed on DCE-MRI images, and the tumor circumference was selected to expand outward 5 mm for semiautomatic profiling, with manual adjustment of the confirmed profiling range. Imaging histology features were extracted from DCE-MRI images of tumor circumference to quantify tumor strength, shape, and texture. In terms of feature selection, the features extracted were selected by using interobserver and intraobserver reliability assessment and LASSO, respectively. The signature of the radiation cohort was constructed from a linear combination of selected features. The performance of the predictive model was assessed by the area under the subject's working characteristic (ROC) curve. To provide a more comprehensible measurement of results, we developed a nomogram personalized assessment tool that evaluates the fitting excellence of column lines by calibrating curves and analyses the clinical utility of column lines by decision curves.

**Figure 2:** Radiomics feature selection by using parametric methods, minimum absolute contraction, and selection operator (LASSO) logistic regression. Intratumora (a-b); periatumoral (c-d); intratumoral combined with peritumoral (e-f).

**Figure 3:** (a) A radiomics nomogram was developed in the training cohort, incorporating the radiomics signature, MR-reported maximum diameter of the lesion, and MR-reported axillary lymph node (ALN) status. Comparison of receiver operating characteristic curves between the radiomics nomogram, intratumoral model, peritumoral model, intratumoral model, intratumoral combined with peritumoral model and model, and MR-reported ALN status alone for the prediction of ALN metastasis in the training (b) and validation (c) cohorts. Calibration curves of the radiomics nomogram in the training (d) and (e) validation cohorts.

**Figure 4:** Analysis of decision curves for each model in the validation dataset. Decision curves show that the use of radiomics models to predict axillary lymph node (ALN) metastasis has additional benefits when the threshold probability exceeds 17% compared to treating all or no patients, intratumoral models, intratumoral models, intratumoral models, and intratumoral combination models.

**Table 1:** Characteristics of patients in primary and validation cohorts.

Characteristic	Training cohort (*n* = 250)			Validation cohort (*n* = 62)		
	Negative for ALN metastasis	Positive for ALN metastasis	*P* value	Negative for ALN metastasis	Positive for ALN metastasis	*P* value
Age	49.171 ± 9.443	47.439 ± 9.697	0.162	52.132 ± 9.062	49.792 ± 11.580	0.378
Max diameter	2.071 ± 0.855	2.283 ± 0.799	0.051	1.853 ± 0.581	2.588 ± 0.852	<0.001
RAD_Sig	0.334 ± 0.0830	0.508 ± 0.135	<0.001	0.344 ± 0.101	0.445 ± 0.120	<0.001
Menopausal state			0.423			0.178
0	90 (0.592)	63 (0.643)		17 (0.447)	15 (0.625)	
1	62 (0.408)	35 (0.357)		21 (0.553)	9 (0.375)	
MR reported _ALN status			<0.001			<0.001
0	131 (0.862)	43 (0.439)		31 (0.816)	9 (0.375)	
1	21 (0.138)	55 (0.561)		7 (0.184)	15 (0.625)	

**Table 2:** Evaluation results of the imaging model in the training cohort and validation cohort.

Performance indicators	Intratumoral		Peritumoral		Intratumoral + peritumoral	
	Training	Validation	Training	Validation	Training	Validation
AUC	0.844	0.708	0.828	0.616	0.867	0.768
Accuracy	0.740	0.677	0.732	0.629	0.768	0.677
Sensitivity	0.714	0.708	0.776	0.500	0.929	0.958
Specificity	0.875	0.757	0.763	0.789	0.651	0.552

## Data Availability

The experimental data used to support the findings of this study can be obtained from the corresponding author upon request.

## Appendix

### Detail Information on the Formula for Intratumoral Combined with Peritumoral radiomics score

Intratumoral radiomics score = 0.3841523939242316++0.002638*∗*lbp-3D-k_glcm_Idn+0.010695*∗*lbp-3D-k_glcm_Imc2+0.051018*∗*lbp-3D-m2_glcm_ClusterShade-0.000916*∗*lbp-3D-m2_glrlm_LongRunHighGrayLevelEmphasis-0.009303*∗*log-sigma-2-0-mm-3D_firstorder_Maximum-0.038417*∗*log-sigma-3-0-mm-3D_firstorder_10Percentile+0.007827*∗*log-sigma-5-0-mm-3D_firstorder_Skewness-0.000488*∗*wavelet-HHH_glcm_InverseVariance-0.020392*∗*wavelet-HHL_firstorder_Kurtosis-0.012501*∗*wavelet-HLH_glcm_Idm-0.021809*∗*wavelet-HLH_glcm_Idn -0.005035 *∗* wavelet-HLL_firstorder_Skewness.

Periatumoral radiomics score = 0.38197102165709085 ++0.004196 *∗*gradient_firstorder_Skewness-0.000437*∗* lbp-3D-k_glrlm_LongRunLowGrayLevelEmphasis-0.003706*∗*log-sigma-3-0-mm-3D_firstorder_Skewness -0.015966 *∗* original_shape_Sphericity -0.020106*∗*square_ glszm_SmallAreaHighGrayLevelEmphasis+0.005082*∗*wavelet-HHL_firstorder_ Skewness -0.012252 *∗* wavelet-LHL_firstorder_Skewness.
